The article "CSF p-tau as a potential cognition impairment biomarker in ALS" was retracted in 2024. Reasons: original data or images not available; unreliable results or conclusions; concerns about the data.

# CSF p-tau as a potential cognition impairment biomarker in ALS

**DOI:** 10.3389/fneur.2022.991143

**Published:** 2022-11-01

**Authors:** Zhongying Gong, Lina Gao, Yi Lu, Zhiyun Wang

**Affiliations:** Department of Neurology, Tianjin First Central Hospital, School of Medicine, Nankai University, Tianjin, China

**Keywords:** amyotrophic lateral sclerosis, cognition impairment, P-tau, T-tau, p-tau:t-tau ratio

## Abstract

**Background:**

Cerebrospinal fluid (CSF) and serum tau (t-tau, p-tau) are potential biomarkers for neurodegeneration in Alzheimer disease (AD), but their role in amyotrophic lateral sclerosis (ALS) is unclear.

**Objectives:**

The aim of our study was to evaluate CSF and serum p-tau and t-tau in patients with ALS and to analyze the correlation and clinical parameters between them.

**Methods:**

CSF and serum samples were obtained from 90 patients with ALS, 48 other neurological disease (OND), and 20 with AM (ALS mimic, AM) diseases. The levels of p-tau and t-tau in the CSF and serum were assessed with an enzyme-linked immunosorbent assay, and disease progression parameters, including the duration, the ALSFRS-R score, disease progression rate (DPR), the upper motor neuron (UMN) score, the Mini-mental State Examination (MMSE) score, the Montreal Cognitive Assessment (MoCA) score, and the Edinburgh Cognitive and Behavioral ALS Screen (ECAS) results, were analyzed by registered neurologists. Statistical analyses were performed using Prism software.

**Results:**

Compared with controls, patients with ALS displayed significantly lower levels of CSF p-tau and p-tau:t-tau ratio. The CSF p-tau level in patients with ALS and cognition impairment was higher than that in patients with ALS who did not have cognition impairment. CSF p-tau level was negatively correlated with MMSE, MoCA, and ECAS total score and the specific score of ECAS in patients with ALS and cognition impairment.

**Conclusions:**

The CSF p-tau level and p-tau:t-tau ratio were lower in patients with ALS than patients with OND and AM. Results suggest that CSF p-tau may be used as an index of cognition impairment in patients with ALS.

## Introduction

Tau protein is one of the main types of proteins in the microtubule-associated protein family. It is a soluble protein and widely expressed in neurons (1). Tau protein can be phosphorylated by specific kinases to form p-tau isomers, resulting in its separation from microtubules; this leads to instability and disintegration (1, 2). Several central nervous system diseases, including Alzheimer disease (AD), encephalomyelitis, and ischemic stroke, show increased level of tau protein in the cerebrospinal fluid (CSF) (3). Increased total tau protein (t-tau) and phosphorylated tau protein (p-tau) in serum and the CSF have been regarded as one of the diagnostic criteria of AD (4). Abnormalities in the CSF and serum tau proteins were found in patients with amyotrophic lateral sclerosis (ALS) in previous studies (5). However, results were not consistent; in the current literature, tau proteins were found to either increase, decrease, or remain stable in patients with ALS (5–7). Abnormal expression of tau protein is closely related to frontotemporal dementia (FTD), Creutzfeldt-Jakob disease (CJD), and AD, and CSF tau protein is closely related to the phenotype for cognitive impairment in progressive supranuclear palsy (PSP) (8). Recent studies have shown that cognitive dysfunction is one of the main symptoms of ALS outside of motor symptoms, with 30–50% of patients experiencing cognition impairment according a current study (9). However, the correlation between tau protein and cognitive function in ALS is still unclear. Previous studies have shown that tau phosphorylated at threonine 181 (p-tau) is pathogenic, changes of p-tau level in ALS from China is unclear. The aim of this study was to investigate changes in CSF and serum p-tau and t-tau levels in a group of Chinese patients with ALS. Furthermore, we analyzed correlations between tau levels, the Mini-Mental Status Examination (MMSE) score, the Montreal Cognitive Assessment Test (MoCA) score, the Edinburgh Cognitive and Behavioral ALS Screen (ECAS) results, the upper motor neuron (UMN) score, disease duration, disease progression rate (DPR), and severity of the disease.

The article "CSF p-tau as a potential cognition impairment biomarker in ALS" was retracted in 2024. Reasons: original data or images not available; unreliable results or conclusions; concerns about the data.

### Materials and methods

This study was a prospective cohort study that biological sample and clinical information were analyzed from the ALS patient database of TFCH. In this study, The OND (other non-inflammatory neurological disease, OND) and AM (ALS mimics, AM) were selected as control who were from inpatients in the same periods. A total of 90 patients who were first diagnosed with *clinically definite* or *clinically probable* ALS according to the modified EI Escorial criteria (10) and who were not taking any medicine were included in this study, as well as patients diagnosed with ALS-FTD had been excluded according to the Rascovsky criteria (11). The patients were diagnosed during the period of January 01 2015, to February 01, 2020, at the Department of Neurology, Tianjin First Central Hospital, School of Medicine, Nankai University. This study was approved by the Ethics Committee of Tianjin First Central Hospital (No: 2018N055KY). After written informed consent was received from all participants, peripheral whole blood was drawn at the time of diagnosis. The cohort consisted of 54 men (60%) and 36 women (40%); 30 of these patients (33%) had ALS onset in the bulbar region of the brain, whereas 60 patients (67%) had onset of symptoms in the limbs. Cognition impairment definited MoCA <26. Disease duration refers to the time from symptom onset to the time of disease diagnosis. The disability level associated with the development and progression of ALS was determined by means of the ALS Functional Rating Scale-Revised (ALSFRS-R) (12) at the time of diagnosis. After enrolling in the study, patients with ALS were evaluated by ALSFRS-R every 6 months, and the difference between the first 6 months and the baseline measurements was calculated and recorded as the decrease in ALSFRS-R score. The DPR (13) was defined as the ALSFRS-R score and disease duration (measured in months). Regarding clinical evaluation, a UMN score of 15 points comprised a number of pathologically brisk reflexes, i.e., abnormal glabellar tap response; facial jerk; jaw jerk; biceps, triceps, finger, knee, and ankle reflexes; and extensor plantar response. The CSF samples were obtained from the patients with ALS and the control patients using lumbar puncture.

The article "CSF p-tau as a potential cognition impairment biomarker in ALS" was retracted in 2024. Reasons: original data or images not available; unreliable results or conclusions; concerns about the data.

A total of 48 age-and sex-matched patients with OND, including tension-type headache (*n* = 38; 79%), hypokalemic paralysis (*n* = 4; 8%), low intracranial pressure (*n* = 1; 2%), and CSF leakage (*n* = 5; 10%) were selected as the control group. This group of OND mainly consisted of non-degenerative diseases. 25 men (52%) and 23 women (48%) with a mean ± SD age of 55.42 ± 11.83 years.

Twenty patients with ALS mimic (AM) diseases served as disease control group, including two patients (10%) with multifocal motor neuropathy, 3 patients (15%) with hereditary spastic paraparesis, and 15 patients (75%) with cervical spondylotic myelopathy. The diagnosis of AM is made by the examination of cervical magnetic resonance imaging, electromyography, cerebrospinal fluid, relative gene detection and so on. All patients were interviewed and examined by neurologists from the study group who had experience with motor neuron diseases.

A blood and CSF sample was collected from the same patient in the control group. All participants enrolled in this study received routine examinations on admission, including hepatic and renal functional assessments. Patients with severe cardiac, liver, or renal dysfunction were excluded.

### CSF and serum sample collection

Blood samples were drawn from all study participants and centrifuged at 3,000g at 4°C for 10 min within 2 h of collection. Supernatants were stored at −80°C until the beginning of the experiment. The mean ± SD time from blood draw to centrifugation was 89.26 ± 32.59 min. The CSF samples were obtained from 48 patients with ALS, 40 patients with OND, and 20 patients with AM disease at the time of diagnosis in our department after lumbar puncture for CSF analysis, the samples were immediately centrifuged at 800g at 4°C for 5 min. Supernatants were stored at −80°C until the beginning of the experiment. The mean ± SD time from lumbar puncture to centrifugation was 85.24 ±17.82 min.

The article "CSF p-tau as a potential cognition impairment biomarker in ALS" was retracted in 2024. Reasons: original data or images not available; unreliable results or conclusions; concerns about the data.

### Enzyme-linked immunosorbent assay for p-tau and t-tau

The ELISA protocol used in this study is as follows: The p-tau181 original Standard reagent was diluted into 0, 0.5, 1.0, 2.5, 5.0, and 10 μg/ml. After preparing reagents, samples and standards, p-tau was added into monoclonal antibody Enzyme wells which are pre-coated with p-tau antibody: 100 μl/well of the standards and 50 μl/well of enzyme conjugate were added into the Standard wells, while 100 μl/well of the samples and 50 μl/well of enzyme conjugate were added into the test wells. After incubated for 60 min at 37°C, the plates were washed five times with the wash solution to remove the uncombined enzyme and then incubated with 50 μl/well of chromogen solution A and 50 μl/well of chromogen solution B for 10 min at 37°C away from light. After incubation, 50 μl/well of stop solution was used to stop the reaction and visualize the reaction products. And the optical density (OD) was measured at a wavelength of 450 nm by a BioTek Synergy 2 microplate reader (BioTek, USA) within 10 min. According to standards' concentrations and the corresponding OD values, the standard curve linear regression equation was calculated out, and then the corresponding samples' concentrations were obtained by applying the OD values of the samples on the regression equation. ELISA for t-tau is the same as p-tau, except the original Standard reagent was diluted into 0, 50, 100, 200, 400, and 800 μg/ml. Non-measurable p-tau or t-tau samples were reported as 0 μg/ml. If required, samples were appropriately diluted to be within the range of the standard curve.

### Statistical analysis

All graphs were generated using GRAPHPAD PRISM, version 7 (Graph Pad Software, Inc.). Normal distributions of data sets were checked using quintile-quintile (Q–Q) plots. One-way ANNOVA analysis were conducted when compared among ALS, OND and AM. Whereas, the results were compared after testing for normal distribution using either the Student *t*-test or Mann-Whitney *U* test when two sets of data are compared. Pearson correlation test was used for statistical correlations between CSF and serum p-tau level, t-tau level, and either MMSE, MoCA, ECAS, UMN, or ALSFRS-R scores, time onset, or the DPR. Statistical data were expressed as the mean ± SE. All *P*-values were 2-sided, and statistical significance was set at *P* < 0.05. Data were analyzed from May 15, 2019, to March 05, 2020.

The article "CSF p-tau as a potential cognition impairment biomarker in ALS" was retracted in 2024. Reasons: original data or images not available; unreliable results or conclusions; concerns about the data.

## Results

### Demographic and clinical characteristics of the patients with ALS and the control patients

There were no significantly differences in age, gender, BMI, BG, Chol, TG, LDL-c, HDL-c and education among ALS, OND, and AM. Details of the patients and controls are summarized in Table 1.

**Table 1:** Demographic and clinical characteristics of the patients with ALS, OND and AM patients ($\bar{x}\pm s$).

	**ALS**	**OND**	**AM**
Cases (*n*)	90	48	20
Age (year)	60.16 ± 12.51	58.42 ± 11.83	59.85 ± 10.24
Gender (M/F)	49/41	25/23	11/9
Specimen (CSF/S)	90/40	48/48	20/20
Education (year)	8.88 ± 4.94	8.83 ± 4.61	9.10 ± 5.40
Definite/probable	46/44	NA	NA
Limb/bulb	53/27	NA	NA
Classic/UMN-ALS/LMN-ALS	49/27/14	NA	NA
ALSFRS-R	35.94 ± 6.98	NA	NA
DPR	1.14 ± 0.80	NA	NA
UMN Score	8.77 ± 0.54	NA	NA
Diagnosis delay (m)	13.26 ± 0.81	NA	NA
BMI (kg/m^2^)	21.90 ± 1.47	21.91 ± 1.78	22.10 ± 1.84
BG (mmol/l)	5.76 ± 2.63	5.67 ± 1.92	5.73 ± 2.24
Chol (mmol/l)	4.84 ± 0.90	4.82 ± 0.88	4.78 ± 0.91
LDL-c (mmol/l)	2.95 ± 0.71	2.93 ± 0.78	2.89 ± 0.74
TG (mmol/l)	1.37 ± 0.76	1.38 ± 0.94	1.41 ± 0.89
HDL (mmol/l)	1.23 ± 0.24	1.24 ± 0.28	1.26 ± 0.27

ALS, amyotrophic lateral sclerosis; ALSFRS-R, ALS functional rating scale-revised; AM, ALS mimic; CSF, cerebrospinal fluid; DPR, disease progression rate; F, female; LMN, lower motor neuron; M, male; OND, other neurologic disease; S, serum; UMN, upper motor neuron. NA, not applicable.

### CSF and serum p-tau and t-tau levels in patients with ALS and control patients

We first examined the levels of p-tau and t-tau in both the CSF and serum. Results indicated that there was no significant difference in CSF t-tau level between patients with ALS (101.30 ± 5.33 pg/mL) and control patients (OND, 105.60 ± 7.59 pg/mL, *P* = 0.8720) and AM (100.20 ± 5.00 pg/mL, *P* = 0.9945), data shown in Figure 1A. There was no significant difference in serum t-tau level between patients with ALS (345.1 ± 5.33 pg/mL) and control patients (OND, 338.3 ± 10.51 pg/mL, *P* = 0.7989; and AM, 341.9 ± 10.44 pg/mL, *P* = 0.9731), data shown in Figure 1B. However, we found that levels of CSF p-tau in the ALS group were significantly different from those in the OND and AM group, as shown in Figure 1C. The CSF p-tau levels in patients with ALS (4.19 ± 0.32 pg/mL) were significantly lower compared with those with OND (23.64 ± 1.49 pg/mL, *P* < 0.0001), the CSF p-tau levels in patients with OND (23.64 ± 1.49 pg/mL) were significantly higher than AM (5.93 ± 0.77 pg/mL, *P* < 0.0001). There was no significant differences in CSF p-tau between ALS (4.19 ± 0.32 pg/mL) and AM (5.93 ± 0.77 pg/mL, *P* = 0.6223). In addition, The serum p-tau level in ALS (51.61 ± 2.32 pg/mL) was lower than that in the OND (57.44± 3.42 pg/mL, *P* = 0.0343), differences were not found in serum p-tau levels between patients with ALS (51.61 ± 2.32 pg/mL) and AM (53.57 ± 3.22 pg/mL, *P* = 0.8123), data shown in Figure 1D.

The article "CSF p-tau as a potential cognition impairment biomarker in ALS" was retracted in 2024. Reasons: original data or images not available; unreliable results or conclusions; concerns about the data.

**Figure 1:** The CSF (*n*_ALS_ = 48, *n*_OND_ = 48, *n*_AM_ = 20) and serum (*n*_ALS_ = 90, *n*_OND_ = 48, *n*_AM_ = 20) p-tau and t-tau level in patients with ALS and control patients. **(A)** CSF t-tau level in ALS, OND, and AM groups; **(B)** serum t-tau level in ALS, OND, and AM groups; **(C)** CSF p-tau level in ALS, OND, and AM groups; **(D)** serum p-tau level in ALS, OND, and AM groups. Statistically analysis was performed with One-way ANNOVA analysis. *P < 0.05 compared with the OND group. ^#^*P* < 0.05 compared with the AM group.

### CSF and serum p-tau:t-tau ratio in patients with ALS and control patients

The ratio of CSF p-tau:t-tau (2.54 ± 0.18, *P* < 0.0001) in the ALS patient group and AM group (5.01 ± 0.70, *P* = 0.0337) was significantly lower than that in the OND group (9.31 ± 1.49). In addition, there was no significant difference in serum p-tau:t-tau ratio among patients ALS (15.3 ± 0.37), OND (16.8 ± 0.63) and AM (15.26 ± 0.52); data shown in Figure 2.

**Figure 2:** The CSF and serum p-tau:t-tau ratio in patients with ALS and control patients. **(A)** CSF p-tau:t-tau ratio in ALS (*n* = 48), OND (*n* = 48), and AM (*n* = 20) groups; **(B)** Serum p-tau:t-tau ratio in ALS (*n* = 90), OND (*n* = 48), and AM (*n* = 20) groups. Statistically analysis was performed with One-way ANNOVA analysis. *P < 0.05 compared with the OND group. ^#^*P* < 0.05 compared with the AM group.

### CSF p-tau and t-tau levels in patients with ALS with and no cognitive impairment

The CSF p-tau level in patients with ALS and cognitive impairment (5.78 ± 0.48 pg/mL, *n* = 18) was higher than that of patients without cognitive impairment (3.17 ± 0.30 pg/mL, *n* = 30; *P* < 0.0001). There was no significant difference in the CSF t-tau level between patients with ALS and cognitive dysfunction (101.30 ± 5.33 pg/mL, *n* = 18) and patients with ALS and no cognitive dysfunction (95.95 ± 8.06 pg/mL, *n* = 30; *P* = 0.9790; Figure 3).

**Figure 3:** Comparison of CSF p-tau and t-tau level in patients with ALS with (*n* = 18) and without cognitive impairment (*n* = 30). **(A)** CSF p-tau level in patients with ALS with and without cognitive impairment; **(B)** CSF t-tau level in patients with ALS with and without cognitive dysfunction. Statistically analysis was performed with Student *t*-test or Mann-Whitney *U* test. ALS-CI, patient with ALS and cognitive impairment; ALS-NonCI, patient with ALS and no cognitive impairment. *P < 0.05, compared with ALS-CI.

The article "CSF p-tau as a potential cognition impairment biomarker in ALS" was retracted in 2024. Reasons: original data or images not available; unreliable results or conclusions; concerns about the data.

### Correlation analysis of CSF p-tau level and cognitive function in patients with ALS

The CSF p-tau level was negatively correlated with MMSE (*r* = −0.4322; *P* = 0.0022), MoCA score (*r* = −0.4906 *P* = 0.0004); data shown in Figures 4A,B. Moreover, there was a negative correlation with ECAS score. Further analysis indicated that CSF p-tau level was negatively correlated with ECAS total score (*r* = −0.5502; *P* = 0.0009), and ALS-specific score (*r* = −0.5412; *P* = 0.0011), especially in *excutive* function (*r* = −0.4583; *P* = 0.0073) and verbal fluency in patients with cognitive impairment (*r* = −0.5525; *P* = 0.0009). However, there was no correlation between CSF p-tau level and language score (*r* = −0.3042; *P* = 0.0852) or ALS non-specific score (*r* = −0.0969; *P* = 0.5963; Figure 4C).

**Figure 4:** Correlation analysis between CSF p-tau and MMSE, MoCA, ECAS total score and each specific score in patients with ALS. Statistically analysis was performed with Pearson correlation test. **(A)** Correlation analysis between CSF p-tau and MMSE. **(B)** Correlation analysis between CSF p-tau and MoCA. **(C)** Correlation analysis between CSF p-tau and ECAS total score and each specific score. Statistically analysis was performed with Pearson correlation test.

### Correlation analysis between ALS CSF and serum t-tau level, p-tau level, disease duration, DRP, ALSFRS-R, survival period, and UMN score

There was no significant correlation between CSF p-tau and t-tau level in patients with ALS and disease duration, DPR, ALSFRS-R score, and survival. There was no significant correlation between serum p-tau and t-tau level in patients with ALS and disease duration, DPR, ALSFRS-R score, and survival. However, CSF p-tau levels in patients with ALS were positively correlated with UMN score (*r* = 0.5279; *P* = 0.0001). In addition, CSF p-tau level in patients with ALS were negatively correlated with UMN score changes at 6 months (*r* = −0.37; *P* = 0.0096; Figure 5).

**Figure 5:** Correlation analysis between CSF p-tau level and UMN score and δUMN score (change of UMN score between the time point of diagnosis and 6 months after diagnosis). **(A)** Correlation analysis between p-tau level in the CSF and UMN score in patients with ALS. **(B)** Correlation analysis between p-tau level in the CSF and δUMN score in patients with ALS. Statistically analysis was performed with Pearson correlation test.

## Discussion

ALS is a heterogeneous group of neurodegenerative diseases that primarily involve the motor system, but cognitive impairment is also an important manifestation of the disease and has received a great deal of attention in recent years (14). The detection of biomarkers in biological fluid specimens is a simple and convenient way to assist in the diagnosis of the disease and to assess prognosis, and is also easily accepted by patients (15, 16). Increased cerebrospinal fluid t-tau and p-tau have been included as one of the diagnostic criteria for AD in the revised International Working Group 2014 (IWG-2) (17). However, there are no consistent results on alterations in cerebrospinal fluid and serum/plasma tau protein in ALS patients (18, 19).

The article "CSF p-tau as a potential cognition impairment biomarker in ALS" was retracted in 2024. Reasons: original data or images not available; unreliable results or conclusions; concerns about the data.

Tau is a microtubule-associated protein that plays a key role in nerve growth (20). Under physiological conditions, phosphorylation of tau provides the necessary kinetic support for neurite formation (8, 21). However, in AD patients, tau phosphorylation levels are two to three times higher than normal and hyperphosphorylation of tau destabilizes tau and microtubules, leading to microtubule instability and transport deficits (22, 23).

In this study, we performed a clinical study on serum and CSF p-tau and t-tau levels in a group of Chinese patients with ALS, which revealed that CSF p-tau level was significantly lower than that of the non-inflammatory OND group. Several studies report alterations in tau phosphorylation in both sporadic and familial ALS (24–26). The decrease of p-tau-T181 in CSF is common, we got similar results in this study. The correlation between p-tau and ALSFRS-r had also been reported, but, it was not confirmed by our results. Some scholars have also found that CSF tau protein increases in the early stage of ALS, with a gradual decline in later stages of the disease (25). The delay in enrollment and diagnosis of patients with ALS may be an additional reason for the decreased level of p-tau (25, 26). There was no correlation between serum and CSF p-tau in patients with ALS in this study, which suggests that the CSF p-tau test may not be explained by serologic detection. However, tau can be phosphorylated at several sites, specific residues of tau phosphorylation in ALS in the brain and spinal cord had been found, such as hyperphosphorylated tau (T175, T217, S208/210, S212, S396, and S404), which were increased significantly in the post-mortem motor cortex and spinal cord of ALS. In addition, ptau-S396 level are increased in C9ORF72-ALS (27). Another study also demonstrated a complexed tau phosphorylated at specific residues (pS396, pS214), which suggest tau phosphorylation plays a role in ALS (28). Therefore, examination of other phosphorylation site might be informative, and it is important to evaluate the gene type of ALS. In addition, a cleavage fragment of tau, Tau_45 − 230_ preceding tau phosphorylation might play a neurotoxic role in the mechanisms of leading to the degeneration of motor neurons in sporadic ALS (29), which is worthy of our concern.

The article "CSF p-tau as a potential cognition impairment biomarker in ALS" was retracted in 2024. Reasons: original data or images not available; unreliable results or conclusions; concerns about the data.

This study also found that the CSF t-tau in patients with ALS was not significantly abnormal compared with that of the control group. Current research suggests that there are no consistent results in the change of CSF t-tau level in patients with ALS, which has been reported as normal in some studies but elevated in others (6, 30, 31). The results of this study differ from previous studies, possibly due to disease heterogeneity, different testing conditions or differences in sample size (32). In addition, our study indicated that the ratio of p-tau:t-tau in the CSF of patients with ALS was lower than that of the control group. Alterations of CSF p-tau:t-tau ratio in ALS have been reported in several studies (6, 30, 31). Our findings also revealed a significant decrease in p-tau-T181:tau ratio in a group of ALS patients from China, which is consistent with previous reports. The above results might indicate the ongoing massive neurodegeneration occurring in the symptomatic phage of ALS. Correlations had been found between p-tau-T181:tau ratio and cognitive function, however, we found no correlation between them, reasons may lie in the differences in race and genetic abnormalities and so on. Thus, the conclusion still need to be verified in a larger sample of ALS from multi-center over the world.

The correlation between CSF and serum tau in ALS patients and clinical parameters such as disease duration, onset, severity and early disease progression was next analyzed. Results suggest that the serum and CSF tau protein were not significantly correlated with these indicators, suggesting that the CSF and serum tau protein may not be not an effective indicator for assessing the progression and prognosis of ALS disease. Previous studies have shown that CSF tau does not significantly correlate with disease duration, disease severity, DPR or disease survival in patients with other types of motor neuron disease and ALS (5, 33, 34), and our results are similar to the above studies. However, we found a positive correlation between CSF p-tau and UMN scores in this group of patients with ALS. Our study results suggest that the increased level of CSF p-tau may reflect UMN damage to a certain extent, which is consistent with previous results (31). The results of the analysis of the correlation between CSF p-tau and cognitive dysfunction in ALS suggest that the CSF p-tau level in patients with ALS and cognitive dysfunction is higher than that of those without cognitive dysfunction. Further analysis suggests that the CSF p-tau level was negatively correlated with MMSE, MoCA, and the specific scores of ECAS in patients with ALS and cognitive impairment, particularly in the area of executive function. The results suggest that CSF p-tau may be closely related to the cognitive function of ALS. Increased CSF tau protein can present in a variety of diseases accompanied by cognitive dysfunction, including AD, PSP, cortical basal ganglia degeneration, dementia with Lewy bodies (DLB), CJD and even in patients with uremia and recognition dysfunction, which was correlated with the severity of the disease and the degree of cognitive dysfunction (35–37). In summary, CSF p-tau protein may be an indicator of cognitive impairment.

The article "CSF p-tau as a potential cognition impairment biomarker in ALS" was retracted in 2024. Reasons: original data or images not available; unreliable results or conclusions; concerns about the data.

In this study, our results showed that CSF p-tau levels and the p-tau:t-tau ratio were decreased in a cohort of Chinese patients with ALS. Our results confirmed the correlation between p-tau level and cognition impairment and UMN score. Because of the small number of enrolled patients, a direct correlation between CSF p-tau level and cognition impairment (including UMN injury) in a broader ALS population could not be established. Future studies should be well designed and include a higher number of ALS patients with defined categories in the EI Escorial criteria from multiple centers. In addition, further genotyping of ALS will help to explore the value of CSF p-tau.

## Conclusion

In this study, we found that the CSF p-tau level and the p-tau:t-tau ratio were lower in patients with ALS. In patients with cognitive impairment, CSF p-tau was negatively correlated with MMSE scores, MoCA scores, total ECAS score, and specific ECAS score, particularly in executive function and verbal fluency. However, there was no correlation found between CSF p-tau level and language score. In brief, the results of this study suggest that CSF p-tau may be considered a potential index of cognitive impairment in patients with ALS. However, several limitations of this study must be kept in mind. Firstly, serum tau levels varied greatly between our study and other studies; our study includes ALS patients from China, and so the natural history and clinical features are quite different between China and Western countries (38). Secondly, other reasons such as enrollment criteria and the potential bias due to the choice of pathologies associated with the control group OND might have contributed to this discrepancy. Thirdly, the small number of enrolled ALS patients may not be representative of the general population. Therefore, more definitive conclusions require well- designed future experiments for confirmation.

The article "CSF p-tau as a potential cognition impairment biomarker in ALS" was retracted in 2024. Reasons: original data or images not available; unreliable results or conclusions; concerns about the data.

## Data availability statement

The raw data supporting the conclusions of this article will be made available by the authors, without undue reservation.

## Ethics statement

The studies involving human participants were reviewed and approved by the Ethics Committee from Tianjin First Central Hospital. The patients/participants provided their written informed consent to participate in this study.

## Author contributions

ZG contributed to the conception of the study and performed the data analyses and wrote the manuscript. LG performed the experiment. YL contributed significantly to analysis and manuscript preparation. ZW helped perform the analysis with constructive discussions. All authors contributed to the article and approved the submitted version.

## Funding

This work was supported by the Tianjin Health Committee (2015KZ035, KJ20143, and ZC20055) and the Chun Technology Fund CF201806 from Tianjin First Central Hospital.

## Conflict of interest

The authors declare that the research was conducted in the absence of any commercial or financial relationships that could be construed as a potential conflict of interest.

## Publisher's note

All claims expressed in this article are solely those of the authors and do not necessarily represent those of their affiliated organizations, or those of the publisher, the editors and the reviewers. Any product that may be evaluated in this article, or claim that may be made by its manufacturer, is not guaranteed or endorsed by the publisher.
